# The Value of Dynamic Contrast-Enhanced Magnetic Resonance Imaging (DCE-MRI) in the Differentiation of Pseudoprogression and Recurrence of Intracranial Gliomas

**DOI:** 10.1155/2022/5680522

**Published:** 2022-07-22

**Authors:** Hui Jing, Xuhong Yan, Junjie Li, Danlei Qin, Ning Zhang, Hui Zhang

**Affiliations:** ^1^College of Medical Imaging, Shanxi Medical University, Taiyuan 030001, Shanxi Province, China; ^2^Department of MRI, The Sixth Hospital, Shanxi Medical University, Taiyuan 030008, Shanxi Province, China; ^3^Department of Endocrinology, Shanxi Provincial People's Hospital, Taiyuan 030001, Shanxi Province, China; ^4^Department of Radiology, First Clinical Medical College, Shanxi Medical University, Taiyuan 030001, Shanxi Province, China; ^5^Intelligent Imaging Big Data and Functional Nano-imaging Engineering Research Center of Shanxi Province, Taiyuan 030001, Shanxi Province, China

## Abstract

**Objective:**

The objective of this study was to determine the value of dynamic contrast-enhanced magnetic resonance imaging (DCE-MRI) in assessing postoperative changes in intracranial gliomas.

**Method:**

A total of fifty-one patients who had new enhanced lesions after surgical resection followed by standard radiotherapy and chemotherapy were collected retrospectively from October 2014 to June 2021. The patients were divided into a pseudoprogression group (15 cases) and a recurrence group (36 cases) according to the pathological results of the second operation or a follow-up of more than six months. The follow-up data of all patients were complete, and DCE-MRI was performed. The images were processed to obtain the quantitative parameters *K*^trans^, Ve, and Kep and the semiquantitative parameter iAUC, which were analysed with relevant statistical software.

**Results:**

First, the difference in *K*^trans^ and iAUC values between the two groups was statistically significant (*P* *<* *0.05*), and the difference in Ve and Kep values was not statistically significant (*P* *>* *0.05*). Second, by comparing the area under the curve, threshold, sensitivity and specificity of *K*^trans^, and iAUC, it was found that the iAUC threshold value was slightly higher than that of *K*^trans^, and the specificity of *K*^trans^ was equal to that of iAUC, while the area under the curve and sensitivity of *K*^trans^ were higher than those of iAUC. Third, *K*^trans^ and iAUC had high accuracy in diagnosing recurrence and pseudoprogression, and *K*^trans^ had higher accuracy than iAUC.

**Conclusion:**

In this study, DCE-MRI has a certain diagnostic value in the early differentiation of recurrence and pseudoprogression, offering a new method for the diagnosis and assessment of gliomas after surgery.

## 1. Introduction

The most common malignant primary brain tumours in adults are gliomas, accounting for approximately half of all primary malignant tumours in the brain and having a high rate of disability and death [1, 2]. Because of the invasiveness of gliomas, it is difficult to completely distinguish the boundaries of the tumour during removal, and the sensitivity of radiotherapy and chemotherapy is not high, so most patients have a poor prognosis. There are many experimental therapies currently under active investigation for patients with recurrence. These include immunomodulatory approaches, such as immune checkpoint inhibitors, tumour vaccines, chimeric antigen receptor (CAR)-modified T-cell therapy, and oncolytic virotherapy. Recently developed immune checkpoint inhibitors such as anti-CTLA-4 (ipilimumab) and anti-PD-1 (pembrolizumab and nivolumab) antibodies have demonstrated clinical efficacy in several solid tumours, with clinical trials for glioblastoma ongoing. Alternating electric field therapy in which a portable device is attached to the scalp and delivers continuous low-intensity alternating electric fields has demonstrated prolonged progression-free and overall survival when used in combination with standard therapy. The device was approved in 2015 for the treatment of newly diagnosed glioblastoma and is expected to change the standard of care [3], the prognosis of intracranial gliomas has improved to some extent, but the situation is still not optimistic [3, 4]. At present, the pathogenesis of gliomas is not clear, so it is one of the most difficult tumours to treat, with high mortality and recurrence rates and a low cure rate. Most patients survive for less than two years and are prone to recurrence and pseudoprogression after treatment [5, 6]. Conventional magnetic resonance imaging (MRI) cannot exactly distinguish the two postoperative conditions, and the pathological preparations of the two are completely different. The pathological mechanism of recurrence involves the proliferation of vascular endothelial cells and tumour angiogenesis, resulting in tumour cell proliferation and constant infiltration of the surrounding tissue, which damages the blood-brain barrier. The pathological mechanism of pseudoprogression involves inflammatory cell proliferation, vascular endothelial damage, cell oedema, demyelination, glial cell proliferation, and destruction of the blood-brain barrier, which usually occur within 3–6 months after surgery. Therefore, the two situations require different treatment methods. Patients with recurrence may require reoperation or change their treatment plan, while patients diagnosed with pseudoprogression need to be monitored by short interval MRI scans, closely, and to support the continuation of currently effective therapy for better clinical outcomes [7, 8]. At present, the most commonly used method of differential diagnosis is histopathology, but this method is invasive and has limitations.

Dynamic contrast-enhanced MRI (DCE-MRI) has a higher spatial resolution and can more accurately evaluate tissue blood perfusion and permeability of new tumour vessels by fitting a two-compartment haemodynamic model. As a noninvasive method, it plays an important role in the diagnosis and treatment of gliomas [9]. Zakhari et al. [10] prospectively compared the diagnostic accuracy of dynamic contrast-enhanced (DCE) and dynamic susceptibility contrast (DSC) in distinguishing tumour recurrence (TR) and pseudoprogression (PSP). Hussain et al. [11] showed that DSC and DCE MRI can distinguish brain tumours and be used to determine the type of brain tumour according to haemodynamic and permeability characteristics. Di et al. [12] indicated that quantitative parameters based on DCE-MRI can be used to evaluate the expression of vascular endothelial growth factor (VEGF) in glioma. Bi et al. [13] studied the antitumour growth and antiangiogenic effects of xanthine in mouse glioma by DCE-MRI. At present, DCE-MRI technology is mainly used for preoperative diagnosis and grading of glioma [14–16]. As for postoperative recurrence and pseudoprogression, previous studies reported [17, 18] more quantitative parameters (Ktrans, Ve, Vp, Kep) of DCE-MRI, but less semiquantitative parameter (iAUC). iAUC as a fast, repeatable, and simple semiquantitative technique converts MR signal to a signal concentration curve and can often be correlated to the underlying physiology in tumours [19].Therefore, in this study, using DCE-MRI technology, quantitative parameters such as *K*^trans^, *V*_e_, and *K*_ep_ and semiquantitative parameters such as the area under the initial curve (iAUC) were measured to analyse the blood flow perfusion and vascular permeability of the microvasculature for early differential diagnosis of recurrence versus pseudoprogression.

## 2. Materials and Methods

### 2.1. Research Object

Fifty-one patients from October 2014 to June 2021 who had new enhanced lesions after surgical resection followed by standard radiotherapy and chemotherapy were included as subjects in this study. The patients were divided into two groups according to the pathological results of the second operation or a follow-up of more than six months: a pseudoprogression group (15 cases), with an average age of 51.25 ± 14.65 years old, and a recurrence group (36 cases), with an average age of 45.33 ± 15.32 years old. There were 32 male patients and 19 female patients in this study, with an average age of 48.29 ± 13.74 years. The inclusion criteria of the study subjects were as follows: (1) after total resection of the brain gliomas, the results of postoperative histopathological examination confirmed that the tumours were brain gliomas classified as grade III and grade IV (according to WHO CNS 2007 standard for classification of gliomas); (2) radiotherapy and chemotherapy were carried out simultaneously after the operation and adjuvant chemotherapy, and there was no residual tumour tissue in MRI before radiotherapy and chemotherapy; (3) after radiotherapy and chemotherapy, the MRI images were reexamined, and there were new enhanced regions; and (4) the follow-up data of imaging examination were complete, and the follow-up time was more than six months. The exclusion criteria were as follows: (1) postoperative pathological examination confirmed that the patient had grade I or grade II gliomas; (2) the images of the patient were not clear; and (3) there was no other intracranial malignant tumour. The experiment used a retrospective design and was approved by the Shanxi Medical University Ethics Committee (2019LL101), and the informed consent requirement was waived due to the retrospective study design.

### 2.2. Diagnostic Criteria

The diagnostic criteria for pseudoprogression of intracranial gliomas are as follows: (1) plain MRI scans and enhanced scans were performed within 2 days after the operation. There was no obvious enhancement in the operation area. During the follow-up, there was enhancement in the operative area; however, the enhanced area decreased or remained unchanged, and the clinical symptoms gradually alleviated. (2) During the follow-up, enhanced lesions appeared in the operative area, which was confirmed as pseudoprogression by the pathology results from the second operation. The diagnostic criteria for postoperative recurrence of intracranial gliomas were as follows: (1) plain MRI scans and enhanced scans were performed within 2 days after the operation. There was no obvious enhancement in the operative area. During the follow-up, there was enhancement in the operative area, the enhancement range was expanded, and the clinical symptoms continued to be aggravated. (2) During the follow-up, enhanced lesions appeared in the operative area, and after the second operation, the pathology results confirmed tumour recurrence.

### 2.3. DCE-MRI Imaging Sequence, Parameter Settings, and Scanning Scheme

In this study, all patients were examined on a Siemens superconductive MRI scanner using a combined head and neck coil. All images were calibrated, and the scanning parameters were consistent. The conventional sequence scanning parameters were as follows: T1 weighted imaging (T1WI) : TR: 108 ms, TE: 24 ms, FOV: 240 × 240 mm^2^, matrix: 256 × 256, layer thickness: 5 mm, layer spacing: 2 mm, NEX 3; T2 weighted imaging (T2WI) : TR: 5090 ms, TE: 91 ms, FOV: 240 × 240 mm^2^, matrix: 256 × 256, layer thickness: 5 mm, layer spacing: 2 mm, NEX 3; and T1 weighted imaging conventional enhanced (T1WI-CE) : TR: 108 ms, TE: 24 ms, FOV: 240 × 240 mm^2^, matrix:256×256, layer thickness: 5 mm, layer spacing: 2 mm, NEX 3. DCE-MRI was scanned with a transverse section T1-twist sequence (TR: 6 ms, TE: 2.35 ms, layer thickness: 3.5 mm, layer spacing: 1.5 mm, FOV: 260 × 260 mm^2^, matrix: 186 × 186, flip angle: 10°). The time resolution was 1.3 seconds for precollecting, and the arterial input function (AIF) was obtained. The contrast agent gadolinium diamine (gadolinium diamine is provided by GE Healthcare, Shanghai, China) was injected through the elbow vein at a speed of 4 ml/s and a total amount of 0.1 mmol/kg in the sixth period (a total of 70 periods), and immediately after, 20 ml of saline chaser was injected at the same rate. The total acquisition time was 6 minutes.

The scanning scheme was as follows: (1) the first scan was within 2 days after the operation and before the start of radiotherapy and chemotherapy, and this scan did not include a DCE-MRI scan; (2) the second scan was within 2 months after the operation after receiving simultaneous radiotherapy and chemotherapy, and this scan included a DCE-MRI scan; (3) after that, reexamination was carried out every three months, and the scan included a DCE-MRI scan; (4) each patient was reexamined at least three times, and the follow-up time was more than 6 months.

### 2.4. Image Processing and Parameter Measurement

The original images were processed with Tissue 4D software on a Siemens postprocessing workstation (the haemodynamic model was the classical Tofts linear two-compartment model), and the corresponding pseudo colour images were obtained. A region of interest (ROI) was set at the level with the most obvious enhancement of the lesion by using the T1WI enhanced image as a reference. When drawing the ROI, cystic changes, necrosis, and calcification were avoided, and the area was controlled within 20–25 mm^2^. Then, in the ROI area, quantitative and semiquantitative parameters, including the values of *K*^trans^, *V*_e_, *K*_ep,_ and iAUC, were measured.

### 2.5. Statistical Analysis

In this study, SPSS 25.0 statistical software was used to process and analyse all data, and *P* *<* *0.05* was considered statistically significant. DCE-MRI haemodynamic parameters are expressed as the mean ± standard deviation. When comparing the differences between groups, if the data had a normal distribution and the variance was homogeneous, a two-sample *T*-test was used; if the data did not have a normal distribution, the rank sum test was used. A receiver operating characteristic curve (ROC curve) of parameters that differed significantly between the two groups was drawn, and the area under the curve, optimal threshold, sensitivity, and specificity were calculated.

## 3. Results

### 3.1. Comparison of Parameters of DCE-MRI Images and Differences between the Two Groups

The *K*^trans^, *V*_e_, *K*_ep_, and iAUC values of the pseudoprogression group were lower than those of the recurrence group, and the differences in the Ktrans and iAUC values were statistically significant (*P* *<* *0.05*). For Ve and Kep values, there was no significant difference between the two groups (*P*＞*0.05*). This is presented in Table 1.

### 3.2. ROC Curve and Diagnostic Efficacy of Parameters with Significant Differences between the Two Groups

ROC curves with parameters with significant differences (*K*^trans^ and iAUC) were drawn (Figure 1), and the sensitivity, specificity, area under the curve, and threshold of Ktrans and iAUC were calculated (Table 2, Figures 2 and 3). The analysis showed that the threshold for iAUC was slightly higher than that for *K*^trans^. The sensitivity and area under the curve of *K*^trans^ were both higher than those of iAUC, and the specificity of *K*^trans^ was equal to that of iAUC, suggesting that *K*^trans^ has higher diagnostic efficacy than iAUC.

### 3.3. Accuracy of *K*^trans^ and iAUC in the Diagnosis of Intracranial Gliomas after Surgery

*K* ^trans^ and iAUC have high accuracy in the diagnosis of pseudoprogression and recurrence of gliomas. The accuracy of *K*^trans^ was 92.16% (13 + 34)/51 × 100%. The diagnostic accuracy of the iAUC value was 86.27% ≈ (11 + 33)/51 × 100%. The diagnostic accuracy of K^trans^ was higher than that of iAUC. This is detailed in Tables 3 and 4.

### 3.4. Image Analysis of Pseudoprogression and Recurrence of Intracranial Gliomas

Follow-up and secondary surgery images of pseudoprogression and recurrence of intracranial gliomas are presented in Figures 4 and 5.

## 4. Discussion

As one of the most difficult malignant tumours to treat, intracranial gliomas have the characteristics of a low cure rate and high mortality and disability rates [17]. Therefore, progress in the diagnosis, treatment, and efficacy monitoring of this disease is important for the treatment and prognosis of intracranial gliomas. Conventional MRI can provide information on the general area of the tumour, but it cannot differentiate postoperative pseudoprogression and recurrence [20]. The treatment of postoperative recurrence and pseudoprogression is very different, pseudoprogression can achieve a good prognosis and overall survival rate without invasive treatment intervention, while recurrence patients must be treated in time to delay the further development of the disease. So, it is very important to distinguish the two. Conventional MRI scan, including plain scan and T1WI contrast-enhanced scan, was the most studied in terms of postoperative recurrence and pseudoprogression [21–24]. Due to the similarities between recurrence and pseudoprogression on conventional MRI, it only can provide information on the general area of the tumour. In this study, DCE-MRI was used to display the tumour functional state and tumour internal microvascular blood flow state through quantitative parameters and semiquantitative parameters and provide histopathological state information to refine and distinguish different types of tumour progression (pseudoprogression or recurrence).

DCE-MRI parameters mainly include quantitative parameters *K*^trans^, *V*_*e*_, *V*_*p*_, and *K*_ep,_ and semiquantitative parameter iAUC. The quantitative haemodynamic parameter *K*^trans^ obtained from DCE-MRI images is the transport constant for the contrast medium from the blood vessel to the extravascular extracellular space (EES). The constant is in direct proportion to the permeability of microvascular endothelial cells and plasma flow. *V*_*e*_ is the volume fraction of EES. Vp is the vascular plasma volume. K_ep_ is the reverse transport constant, which is the rate constant of the contrast agent entering the blood vessel from the EES. It can be calculated according to the following equation: *K*_ep_ = *K*^trans^/*V*_*e*_ [25, 26]. The semiquantitative parameter iAUC is the area under the initial curve, which is the change in the signal intensity of the contrast agent in blood vessels and tissues with time, so it can represent the blood volume [27]. It can be seen from the results of this study that the values of *K*^trans^ and iAUC in the pseudoprogression group were lower than those in the recurrence group. The reason may be that pseudoprogression after surgery mainly includes tissue inflammatory reactions, intracellular dermatitis injury, glial cell demyelination, and other injuries, leading to local surrounding tissue oedema and destruction of the blood-brain barrier. The local blood volume is slightly increased, while there is a large amount of tumour cell proliferation, neovascularization, active tissue metabolism, and a large increase in blood volume after recurrence. Through rat model experiments, Du et al. [28] demonstrated that DCE-MRI can be used to evaluate the angiogenesis of glioma. The values of *K*^trans^ and *K*_ep_ are in direct proportion to the amount of angiogenesis, while the values of *V*_*e*_ are in inverse proportion to the amount of angiogenesis, which is basically consistent with the results of this study. Van Dijken et al. [29] showed that the pharmacokinetic parameters *K*^trans^ and iAUC in the recurrent group were higher than those in the pseudoprogression group (*P* *<* *0.01*), which is the same as the results of this study. In this study, the sensitivity and specificity of *K*^trans^ for the diagnosis of recurrence and pseudoprogression were 94.4%, 100%, and the area under the curve was 0.978, while the corresponding values of iAUC were 88.9%, 100%, and 0.900, respectively. This shows that the diagnostic efficacy of this study is higher than that in the previous literature mentioned (*K*^trans^ had a 69% sensitivity and 79% specificity for disease progression, and *K*^trans^ had a 92% sensitivity and 85% specificity for true progression, respectively) [17, 29]. At the same time, the accuracy of *K*^trans^ and iAUC values was calculated in this study, However, there is no report about the accuracy in the previous reference [17, 18].

Through the diagnosis of postoperative progression of intracranial gliomas with these DCE-MRI parameters, the results show that *K*^trans^ and iAUC are valuable. However, the current study has several limitations. First, the study population was relatively small. Second, in the actual clinical treatment process, due to the changes in tumour tissue, as well as the injury associated with surgery, and the effect of radiotherapy and chemotherapy [7, 30, 31], the surgical area is generally complex, so there will be a certain misdiagnosis rate when the diagnosis is based on DCE-MRI alone. Third, the DCE-MRI scan time was relatively long. Fourth, the retrospective study design could cause some selection bias [32]. Therefore, it is necessary to increase the sample size and include other functional magnetic resonance imaging methods to conduct further studies. Prospective studies are also needed to validate the clinical usefulness of our findings and investigate the optimal scanning protocol.

## 5. Conclusion

This study comprehensively analysed the value of DCE-MRI-related parameters in diagnosing recurrence and pseudoprogression of glioma and found that the difference in *K*^trans^ and iAUC values was statistically significant, and their area under the ROC curve, accuracy, sensitivity, and specificity were high, offering a new method for the diagnosis and assessment of gliomas after surgery.

## Figures and Tables

**Figure 1:** ROC curve of K^trans^ and iAUC.

**Figure 2:** Histogram of the sensitivity and specificity of *K*^trans^ and iAUC.

**Figure 3:** Histogram of the area under the ROC curve and threshold of *K*^trans^ and iAUC.

**Figure 4:** Patient, female, 40 years old, left temporal glioma (WHO grade III). (a) The T1WI-CE scanning image before surgery; (b) a T2W1 scanning image 2 days after operation; (c) a T1W1-CE scanning image 2 days after operation; (d) the T2WI scanning image after 12 months of synchronous radiotherapy and chemotherapy; (e) the T1WI-CE scanning image after 12 months of synchronous radiotherapy and chemotherapy; (f) the *K*^trans^ pseudo colour image after 12 months of synchronous radiotherapy and chemotherapy; (g) the iAUC pseudo colour image after 12 months of synchronous radiotherapy and chemotherapy; (h) the T1W1-CE scanning image after 25 months, diagnosed as pseudoprogression of the left temporal glioma.

**Figure 5:** Patient, male, 23 years old, left frontal glioblastoma (WHO grade IV). (a) The preoperative T1WI-CE scanning image; (b) the T2W1 scanning image 2 days after the operation; (c) the T1W1-CE scanning image 2 days after the operation; (d) the follow-up T2W1 scanning image 11 months after the synchronous radiotherapy and chemotherapy; (e) the follow-up T1WI-CE scanning image 11 months after the synchronous radiotherapy and chemotherapy; (f) the *K*^trans^ pseudocolour image after 11 months of synchronous radiotherapy and chemotherapy; (g) the iAUC pseudocolour image 11 months after the synchronous radiotherapy and chemotherapy; (h) the histopathological results (HE ×400) of the second operation, confirming the recurrence of the left frontal glioma.

**Table 1:** Comparison of DCE-MRI parameters in the two groups of patients.

Group	*K * ^trans^ value (min^−1^)	*V *_*e*_ value (%)	K_ep_ value (min^−1^)	iAUC value (mM/s)
Pseudoprogression group	0.0940 ± 0.0155	0.2929 ± 0.0808	0.4469 ± 0.0999	0.1398 ± 0.0297
Recurrence group	0.2728 ± 0.0924	0.3677 ± 0.1387	0.5180 ± 0.1712	0.3210 ± 0.1322
T value	11.244	1.948	1.846	7.763
*P* value	<0.001	0.057	0.072	<0.001

**Table 2:** Results of ROC curve analysis of K^trans^ and iAUC.

Parameter value	Sensitivity (%)	Specificity (%)	Area under the ROC curve	Threshold
*K * ^trans^	94.4	100	0.978	0.1302
iAUC	88.9	100	0.900	0.1929

**Table 3:** Comparison of the results of *K*^trans^ in the diagnosis of intracranial gliomas and pathological diagnosis or follow-up results.

*K * ^trans^ diagnosis	Pathological diagnosis or follow-up results	
	Pseudoprogression group	Recurrence group
Pseudoprogression group	13	2
Recurrence group	2	34
Total	15	36

**Table 4:** Comparison of the iAUC results in the diagnosis of intracranial gliomas and pathological diagnosis or follow-up results.

iAUC diagnosis	Pathological diagnosis or follow-up results	
	Pseudoprogression group	Recurrence group
Pseudoprogression group	11	3
Recurrence group	4	33
Total	15	36

## Data Availability

The datasets used and/or analysed during the current study are available from the corresponding author on reasonable request.
